# Action Recognition, Tracking, and Optimization Analysis of Training Process Based on the Support Vector Regression Model

This article has been retracted.

**DOI:** 10.1155/2022/2174240

**Published:** 2022-03-22

**Authors:** Mingjiang Zhu

**Affiliations:** Department of Physical Education, North China University of Water Resources and Electric Power, Henan 450046, Zhengzhou, China

## Abstract

In order to study the action recognition, tracking, and optimization of the training process based on the support vector regression model, a method of human action recognition based on support vector machine optimization is proposed. This method uses the improved strategy of support vector machine to realize the action recognition through the human action recognition based on the optimization of the vector machine. During the recognition, the DAG SVM strategy is improved according to the recognition accuracy of the classifier, and when outputting the result, output the recognition result and the corresponding confidence level, and use the confidence level to process the recognition result. Finally, through the experimental results, it is realized that the recognition rate based on support vector optimization is 98.7%, indicating that this method is effective and can improve the accuracy and efficiency of human body action recognition.

## 1. Introduction

Human motion recognition is an important research topic in the field of computer vision. It has a certain application prospect in video surveillance, intelligent security, human-computer interaction, virtual reality, and artificial intelligence [1]. Video-based human motion recognition technology is an important part of the human body recognition process, it uses the representation of actions to realize human action recognition based on machine learning methods. Gesture recognition is the basis of human action recognition and two methods are generally used. One is to use sensors to make accelerometers that can be worn on the body or tension sensors that can be installed on clothes; this kind of sensor is more accurate and direct, but it restricts the movement of the limbs, and it is very inconvenient to carry, which will cause a certain burden for users [2]. The other is through a visual capture technology, such as static images or video surveillance images, which uses processing visual data to extract available information and makes judgments on human movements, it mainly expresses the posture characteristics through the body contours, but the contour feature is to describe the posture through the angle of the human body; however, the changes in the details of each part of the body are ignored, and the posture of the human body cannot be accurately determined. Related research studies show that based on the expression of body posture, the human body includes multiple body parts, such as the trunk, neck, and legs [3]. These posture features are all extracted through two-dimensional color images, it is necessary to improve the effects of human body positioning, different light, and body occlusion on recognition. Human action recognition should be based on gesture recognition and relevant human body recognition research must be concentrated in three aspects, including human body posture structure, moving target tracking, and other human action recognition. Studies have shown that Sattari. M. T. proposed human action recognition based on a machine-learning SVM method. In the classification, the SVM classification method is mainly used to perform the time interval feature extraction on the acceleration signal and select the classifier by confidence when training the classifier; finally, all classifiers are called during recognition [4]. Sattari. M. T. proposed an induction motor fault diagnosis based on recursive non-decimated wavelet packet transform and DAG SVM. When it is classified, it mainly compares one-v-all (OVA), one-v-one (OVO), and directed acyclic graph (DAG) [4]. Stefanos G. et al. proposed a 5-parameter MD-H model to improve the singular problem when two adjacent joints of the D-H model are parallel. In terms of measurement, laser trackers, visual tracking systems, and ball bars can achieve high-precision measurements and provide standard quantities for error correction [5, 6].

Based on the literature [7], the supervised learning method based on support vector machine (SVM) is directly introduced, a UP-OP strategy is proposed, which extracts features from the acceleration set and then generates a classification model by optimizing the best parameters, then uses the improvement strategy of DAG SVM to test and identify, output classification results and confidence, and judge the results, so as to achieve efficient and accurate recognition.

## 2. Experimental Analysis

### 2.1. Data Collection

In the research of this article, the linear acceleration (acceleration sensor) database used is the SCUT-NAA database, which is collected by the human-computer intelligent interaction laboratory. The database is the data collected by only one 3D acceleration sensor under completely natural conditions. In the process of human movement, different parts of the body have different movement states. Chavarriage et al. conducted a study on the offset of the position acceleration signal characteristics when the sensor is changed. It is concluded that the wearing part of the detection device should be selected to be a part that changes significantly during exercise but has small acceleration changes in daily life. The quality of the chest position is more concentrated, and the activities in daily life are not frequent; therefore, the data of the coat pocket close to the chest are selected, and the data of the first forty collectors among them are selected to verify the algorithm of this article.

### 2.2. Experimental Process

In order to show the performance of the algorithm in identifying various actions, six different actions are considered: “walk”, “stand”, “run”, “jump”, “upstairs”, and “downstairs”. In order to evaluate the performance of the action, two case studies were conducted: ①Train the actions of all testers and then test and identify the actions of each tester. In the 2 sets of data for each action, the former group is used to train the classifier, and the latter group is used to test the algorithm. The possible “universality” of this test can be used to train a large test group. ② Divide the experimenters into two groups, train the two groups separately, and then use the models obtained by each training to recognize the actions of the other group of testers. In the two sets of data for each action, the first set of data of the two sets is used to train the classifier, and the second set of data is used for the test recognition of the other set of actions. In the test, as shown in Figure 1, the root node of this article selects the static and running classifiers, and the distribution of the entire improved DAG strategy.

### 2.3. Experimental Results

The evaluation of the test result is carried out by comparing the actual action of the tester with the recognized action, if the recognized action is the same as the actual action, then the recognition result is recorded as a correct recognition result; conversely, if the recognized action is not the same as the actual action, then this recognition result is considered to be an erroneous recognition result.  Table 1 shows the test results of the case one scheme. In case one, the test result shows that after the classifier trained by all tester training samples performs test recognition on all test samples, the recognition results of two samples are wrong recognition. Then, after testing and identifying, all test samples according to the UPOP strategy, all samples are identified.

Table 2 shows the test results of the second scenario. In case two, the test results show that the classifier obtained after grouping training with all testers' training samples will test all test samples in groups, the recognition results of thirteen samples are wrong recognition. After testing and identifying, all test samples according to the UP-OP strategy, there are still four samples that cannot be identified.

Through the data shown in Tables 1 and 2 it can be intuitively reflected that the method in this paper has a significant improvement compared to the previous method. After careful analysis, the reason for the wrong recognition result is found to be that the trainer has changed the speed during training and at the same time, the time scale has also changed when the acceleration data is processed; these two reasons lead to the occurrence of misidentification.

## 3. Discussion

### 3.1. Improvement and Optimization of Identification Methods

In order to recognize the daily actions of the human body, the method is based on supervised learning that needs to be trained to recognize actions. First, discuss the classification method used. Then, explain the methods used in human body motion recognition at each stage. Finally, describe and provide detailed algorithms for identifying actions. In the training phase, use the Libsvm toolkit to obtain the optimal training model for the training samples, that is, the optimal C parameter and *g* parameter are obtained under the RBF kernel function, that is, cross-validation is used to automatically search for the optimal parameters *c* and *g*. In the motion recognition stage, the classifier obtained by SVM algorithm training is used. This method is DAG SVM.

The advantage of this classification is that if the number of categories is *k*, only k-1 is called, the classification speed is fast, and there is no classification overlap and non-classification phenomenon. However, there is a serious problem in the DAG strategy, that is, the arrangement order of DAG SVM nodes is irregular, and the arrangement order of different nodes will lead to different paths identified by some samples; this affects the accuracy of recognition. DAG. The closer the classification error occurs to the root, the worse the classification performance; therefore, the most important thing in the DAG strategy is the selection of the root node and it is best to have very different actions [8]. In the testing phase, use the model strategy to test the samples to be tested, and obtain the distance *d*(*x*_*i*_) from each sample *x*_*i*_ to the optimal classification surface of the SVM, that is, the confidence level of each sample to be tested, and the classification result of each test sample. The concept of confidence is introduced here. For each general vector *x*, its confidence is defined as the distance from the hyperplane (*w*, *b*)

(1) $$\begin{array}{c} d\left(w,b;x\right)=\frac{w\cdot x+b}{\left\|w\right\|}. \end{array}$$

This distance is *d*(*w*, *b*; *x*), it shows how confident this classifier is for this vector mushroom type. According to the statistical 3sigma control standard, 95% is used as the commonly used confidence standard. If the rejection confidence threshold *p* is given, the classification result of the sample to be tested with the recognition confidence less than the threshold should be rejected [9]. For the sample rejected for identification, first take the inversion and then output the test identification result. After the statistics and analysis of the final result, the accuracy of the method can be verified.

The standard deviation can reflect the degree of dispersion of sensor acceleration data, and the standard deviation is an important feature that can identify static and dynamic actions. The kurtosis of the *Y*-axis can effectively distinguish running from other types of sports. The skewness of the *X*-axis can effectively distinguish descending stairs from several other actions. The correlation coefficient of *Y*-axis and *Z*-axis can effectively distinguish walking and going upstairs.

Standard deviation: the definition of standard deviation is as follows:

(2) $$\begin{array}{c} \sigma =\sqrt{\frac{1}{\left(N-1\right)}\sum_{i=1}^{N}{\left(X_{i}-\bar{X}\right)}^{2}}. \end{array}$$

In the formula, IV is the number of samples, Ge is the average of the samples, the standard deviation can reflect the degree of dispersion of the sensor acceleration data, standard deviation is an important feature that can identify static and dynamic actions.

The whole process is defined as an UP-OP strategy, which is briefly described as follows.

Input: training sample set, test sample set, rejection confidence threshold *θ*.

Output: test sample classification result decisioni_i_ and sample classification result decisioni_ii_ after rejection recognition processing.

**Step 1 .**

train the samples in the training set samples to obtain the optimal training model.

**Step 2 .**

Improve the DAG SVM strategy.

**Step 3 .**

sequentially test the samples in the sample set to be tested, obtain the classification result decisioni_i_ of the sample to be tested, and the confidence level *d*(*x*_*i*_) of the sample to be tested *x*_*i*_.

**Step 4 .**

Given the rejection confidence threshold *θ*, accept samples with confidence greater than *θ*, directly output the classification result decisioni_i_ of these samples, refuse to identify the rest of the samples, and release the sample set.

**Step 5 .**

Invert the classification result decisioni_i_ of the samples in the rejection sample set and output the test result decisioni_ii_.

**Step 6 .**

Perform statistics and analysis on all results.

### 3.2. Support Vector Machine Regression Model

Support vector machine regression is a machine learning algorithm based on a statistical learning theory. It has a strict mathematical theory foundation, intuitive geometric explanation, and good generalization ability. It has unique advantages in dealing with small sample learning problems, especially suitable for non-linear regression data processing. Given the training set,

(3) $$\begin{array}{c} T=\left\{\left(x_{1}.y_{1}\right),\left(x_{2},y_{2}\right)\cdots \left(x_{m},y_{m}\right)\right\}\in {\left(R^{n},R\right)}^{m}. \end{array}$$

First, the input variables should be mapped from *n* dimensional to *l* dimensional feature space *R*^*n*^⟶*R*^*l*^, *x*⟶*ϕ*(*x*), an optimized hyperplane is constructed in the feature space, and the non-linear problem is transformed into a linear problem.

(4) $$\begin{array}{c} f\left(x\right)=W\phi \left(x\right)+b. \end{array}$$

In the formula, *W* is the *l* dimensional weight vector and *b* is the bias term.

When calculating with SVR, the insensitive loss function measurement of parameter *ε* will be introduced, as shown in formula (5). If the regression function error is less than the loss parameter *ε*, ignore the impact on the regression result and include as many data points as possible.

(5) $$\begin{array}{c} e\left(f\left(x\right)-y\right)=\left\{\begin{array}{c} 0,\left|f\left(x-y\right)<\varepsilon \right|\\ \left|f\left(x\right)-y\right|-\varepsilon \end{array}\right\}. \end{array}$$

By choosing a suitable kernel function, not only can the accuracy of the prediction model be improved but can also reduce the influence of random noise on the prediction model and the amount of calculation. Currently, the commonly used kernel functions and their characteristics are as follows: polynomial function, the computational complexity increases when the dimensionality is too high; linear function, suitable for training models with the same input and output dimensions; the sigmoid function, similar to the structure of a multilayer neural network, has certain limitations; Radial Basis Function (RBF) has low sample requirements, wide application, and high flexibility [10]. Due to the different dimensions of robot input and output and the high complexity of the model, RBF is selected for training, the specific expression is

(6) $$\begin{array}{c} K\left(x,x^{\prime }\right)=\exp\left(-\frac{{\left|x-x\right|}^{2}}{2\sigma^{2}}\right). \end{array}$$

Through the exponential relationship, the input sample space is mapped to the infinite dimensional space, so as to achieve high-precision non-linear fitting.

In order to improve the training accuracy of the SVR model and reduce the influence of nonstructural parameters, it is necessary to divide the robot workspace. The quality of grid division will directly affect the accuracy and speed of robot calibration. The size of the grid is inversely proportional to the calibration result within a certain range. The smaller the grid, it brings great difficulty to the actual operation; the larger the grid, the worse the calibration result.

The meshing steps are as follows:

1. Define grid properties, including shape and size. If the fan-shaped meshing method is used, combining the robot's 3 basic corners for division, this method is more suitable for the robot's movement mode. However, the solution prediction error is in the Cartesian coordinate system, which causes the calibration effect to be unsatisfactory. In view of the above situation, it is convenient for the final error correction and the calibration effect is better. The choice of the cube size is mainly based on the required accuracy. According to the analysis center selected by Hong Peng et al. on the grid size, the UR5 robot is divided into a grid using a 100 mm×*i*00 mm × 100 mm square cube structure.
2. Divide the grid to obtain the sampling point set. The working space of the robot is a sphere, and the grid is divided into a cube structure, it is not possible to cover all spaces. For boundary spaces, minimize the grid size to achieve accurate correction. In a single grid, the effect of the number of sampling points on the final training result is shown in Figure 2. The standard deviation drops rapidly in 0410 sampling intervals, and an inflection point appears in the 10–30 sampling intervals, and the effect of correcting the error tends to be stable. On the premise of ensuring the training results, using fewer training samples can reduce the difficulty of sampling and avoid overfitting. Therefore, 20 points are selected as the sampling number of a single grid.

## 4. Conclusion

It is necessary to comprehensively analyze the advantages and disadvantages of behavior recognition methods. Therefore, this paper proposes a human motion recognition algorithm based on support vector machine optimization. Through the processing of the results and the optimization and improvement of the process, the accuracy and efficiency of motion recognition can be effectively improved. It has certain results in the proposed action recognition algorithm, but there are still areas that need to be improved and improved, so in the future, it is necessary to conduct in-depth research on human motion recognition algorithms. Based on the support vector machine optimization method, by improving and optimizing the recognition process and result processing, in this way, the efficiency and accuracy of action recognition can be improved. The results show that the accuracy of this algorithm for action recognition is 98.3%. The next step will optimize the algorithm of action recognition and strengthen the system training to adapt to other daily actions. Using the feedback from the action recognition stage, the results can be processed through the feedback. In addition, we can also deduce whether it is more convenient to try to use the sensor's orientation (quaternion) instead of only using acceleration data, and the use of forest time series for feature extraction and classification.

## Figures and Tables

**Figure 1:** Strategy based on support vector machine optimization.

**Figure 2:** Relationship between training sample size and calibration accuracy.

**Table 1:** Experimental results of case 1.

Group	Action	Sample	No optimization results (%)	The result after optimization
	Static	50	75	97.2%
	Go	50	100	100%
	Run	50	100	100%
	Jump	50	90	100%
	On	50	100	95%
	Down	50	95	98%
Total			92.1	98.3%

**Table 2:** Scheme test results of the second case.

Group	Action	Sample	No optimization results (%)	The result after optimization (%)
	Static	50	100	100
	Go	50	98	100
	Run	50	97	100
	Jump	50	100	100
	On	50	100	100
	Down	50	100	100
Total			100	100

## Data Availability

The data used to support the findings of this study are available from the corresponding author upon request.
